# Risk Factor Analysis and Construction of a Prognostic Model after Percutaneous Coronary Intervention in Patients with Chronic Total Occlusion

**DOI:** 10.1155/2022/9902380

**Published:** 2022-02-01

**Authors:** Xia Zhao, Xian Yuan, Yi Zhong, Gang Wang

**Affiliations:** ^1^Department of Cardiovascular Medicine, The Second Affiliated Hospital of Jiaxing University, Jiaxing 314000, China; ^2^Department of Cardiology, The Affiliated Huai'an Hospital of Xuzhou Medical University, The Second People's Hospital of Huai'an, Huaihai, Jiangsu Province 223001, China; ^3^Intensive Care Unit, The Affiliated Huai'an Hospital of Xuzhou Medical University, The Second People's Hospital of Huai'an, Huaihai, 223001 Jiangsu Province, China; ^4^Geriatrics Department, Lianshui County People's Hospital, Lianshui County, Huai'an, Jiangsu Province 223400, China

## Abstract

**Methods:**

The clinical data of 82 patients with CTO who underwent PCI in Lianshui County People's Hospital were collected in this study. The patients were divided into training set (*n* = 54) and validation set (*n* = 28) by random sampling method. Statistical difference test was performed for clinical features of patients. Univariate and multivariate Cox regression analyses were performed to determine the risk factors affecting progression of CTO. Nomogram was used to construct a prediction model for disease progression. *C*-index was calculated, and the accuracy of the model was tested by calibration curve.

**Results:**

No statistically significant differences were incorporated in baseline characteristics of included patients (*p* > 0.05). There were 25 patients with adverse cardiac events during follow-up in the training set and 13 in the validation set. The results of multivariate Cox regression analysis demonstrated that the important factors affecting postoperative disease progression mainly came down to age, BMI, diabetes, creatinine clearance rate, and left ventricular fraction < 40%. A nomogram was constructed and *C*-index was calculated. The calibration curve was then used to evaluate and predict risk model of disease progression. The result showed an internal validation *C*-index of 0.6219 and an external validation *C*-index of 0.6453, which indicated the good prediction performance of the model.

**Conclusion:**

The risk of disease progression in CTO patients treated with PCI can be effectively predicted by the risk model constructed in this study, which opens up a great possibility for enriching the means of predicting the prognosis of these patients in clinical practice.

## 1. Introduction

Chronic total occlusion (CTO) is a common complex lesion of the coronary artery which was occluded for ≥3 months with the absence of any forward flow beyond a coronary occlusion (TIMI 0 grade) [1]. Previous studies have found that 20% of patients with coronary heart disease complicate at least one CTO lesion simultaneously [2]. Percutaneous coronary intervention (PCI) is called the “last fortress” in the field of coronary intervention because of its low success rate of surgery and high incidence rate of complications [3]. The efficacy of PCI for CTO can relieve angina pectoris [4], improve left ventricular function, reduce the probability of undergoing coronary artery bypass grafting (CABG), and improve the medium- and long-term survival rate of patients [5]. Several observational studies in China indicate that CTO patients have a better clinical prognosis after PCI treatment. It has been found in 15% to 30% of patients that PCI does help enormously in many aspects such as distal occlusion alleviating, blood supply restoring in supply area, myocardial ischemia improving, and angina pectoris relieving [6]. Coronary occlusion usually lasts for a long time in patients with CTO. Due to the continuous formation of thrombus in atheromatous plaques after coronary artery lesions, the coronary artery is gradually narrowed and occluded by the mixture of proliferating fibrous endothelium and thrombus. The process that occurs slowly may be accompanied by the formation of collateral circulation [7].

The emergence of CTO results from a variety of risk factors including sex, hypertension, smoking, and diabetes [8]. After PCI in patients with CTO, multiple risk factors can exert an effect on the prognosis of patients, which may increase the incidence of adverse cardiovascular events [8]. During clinical treatment, the control of various risk factors of patients should be strengthened to reduce the influence of risk factors. Effective control should be achieved by regular follow-up after patients are discharged from the hospital, thus improving patients' prognosis and their quality of life [9].

In this study, we collected the clinical features of CTO patients treated by PCI. Then, we constructed a risk-proportional regression model and analyzed the clinical risk factors affecting the prognosis of patients. Finally, we discussed the accuracy of this model in predicting the prognosis of patients, with a hope to enrich the means of clinical prediction of prognosis.

## 2. Materials Methods

### 2.1. Study Subjects

This study collected 82 CTO patients admitted to Lianshui County People's Hospital, from July 2018 to December 2019. CTO is defined as the lesion lasting for 3 months with a TIMI blood flow grade of 0. All patients underwent successful PCI with complete clinical information, and patients with major underlying diseases were excluded. This study has been approved by the Ethics Committee of the Lianshui County People's Hospital without patients' informed consent, because the study was merely a retrospective study where clear personal information is not mentioned.

The collected patient samples were divided into training (*n* = 54) and validation (*n* = 28) sets according to the random number method. The risk model was constructed using the training set, and the validation set was used to verify the degree of fit of the constructed model.

The age distribution of patients in the training set was 27 cases ≤ 57 years old and 27 cases > 57 years old (27 cases), involving 22 male and 32 female, and the mean body mass index (BMI) was 24.74 ± 3.40. The age distribution of the patients in the validation set was 47 cases ≤ 57 years old and 13 cases > 57 years old, involving 13 male and 15 female, and the mean BMI was 24.68 ± 2.77. There were no remarkable statistical differences in baseline information between patients in the two groups (Table 1).

### 2.2. Primary Endpoints

The follow-up time of this study was once every three months within one year after enrollment and once every six months in the second and third years. The disease progression status of the patients was determined by regular blood examination, routine urine examination, and renal function examination. Patients and their families were also asked whether there was an occurrence of cardiac adverse events, and the time and frequency of cardiac adverse events were recorded. Cardiac adverse events include cardiac death, congestive heart failure, recurrent angina, nonfatal remyocardial infarction, serious arrhythmia, and re-revascularization.

The outcome measure of this study was the progression of CTO patients after PCI intervention, and the censored data were no disease progression in patients or loss to follow-up at the end of this study.

### 2.3. Statistical Analysis

SPSS 26.0 software was used for testing the statistical difference of clinical features between the two groups. *T* test was used for comparison of measurement data conforming to normal distribution and chi-square test for comparison of enumeration data. Univariate and multivariate Cox regression analyses were performed using the “rms” package of R language. Then, nomogram was constructed. *C*-index was calculated, and the fit of the constructed model was tested using calibration curves. The level of statistical significance in this study was defined as 0.05.

## 3. Results

### 3.1. Univariate Cox Regression Analysis

Univariate Cox regression analysis was performed with all clinical features of patients as influencing factors (Table 2), and the result showed that age (*p* < 0.001) (HR: 1.086, 95% CI: 1.035-1.139), creatinine clearance rate (*p* = 0.022) (HR: 0.954, 95% CI: 0.916-0.993), left ventricular ejection fraction (*p* < 0.001) (HR: 0.860, 95% CI: 0.793-0.931), and diabetes (*p* < 0.001) (HR: 4.269, 95% CI: 1.836-9.927) were implicated in the risk of disease progression in CTO patients.

### 3.2. Multivariate Cox Regression Analysis

Age, BMI, diabetes, creatinine clearance rate, and left ventricular ejection fraction were included in multivariate Cox regression analysis (Table 3). The analysis results showed that age (*p* = 0.006) (HR: 1.113, 95% CI: 1.023-1.092), BMI (*p* < 0.001) (HR: 1.290, 95% CI: 1.081-1.440), diabetes (*p* = 0.047) (HR: 2.873, 95% CI: 0.916-9.685), creatinine clearance rate (*p* = 0.008) (HR: 0.935, 95% CI: 0.899-0.987), and left ventricular ejection fraction (*p* < 0.001) (HR: 0.857, 95% CI: 0.781-0.924) after PCI in patients with CTO were independent factors affecting disease progression.

### 3.3. Nomogram Construction as well as Internal and External Validation

According to the results of multivariate Cox regression analysis, age, BMI, diabetes, creatinine clearance rate, and left ventricular ejection fraction were included as influencing factors to construct a nomogram (Figure 1). And each influencing factor corresponded to a score, and the total score mapped to the axis of progression risk, which could reflect the risk of disease progression in CTO-PCI patients at one and two years.

The accuracy of the model was tested by internal and external validation of the training and validation sets through calibration curves and *C*-index values (Figures 2 and 3). The results showed that the *C*-index of internal validation was 0.6219 and that of external validation was 0.6453, which indicated that the model could better predict the risk of disease progression in CTO patients after PCI.

## 4. Discussion

A large number of studies have discovered that patients with coronary heart disease are prone to adverse cardiovascular events within 1 year after PCI, which greatly affects the prognosis of patients [10, 11]. And the occurrence of adverse cardiovascular events is closely associated with the risk factors of coronary heart disease in addition to their own dietary habits and living habits [12]. In this study, we constructed a risk prognostic model which demonstrated that age, BMI, diabetes, creatinine clearance rate, and left ventricular ejection fraction of CTO patients after PCI may all contribute to the deterioration of adverse cardiovascular events. The internal and external validation of the constructed model was performed by *C*-index. The results illustrated that the *C*-index of internal validation was 0.6219, and the *C*-index of external validation was 0.6453. This model successfully predicted the progression of cardiovascular adverse events after PCI, which enriched the means of clinical prediction of the prognosis of these patients. There were 25 cases of adverse cardiac events during follow-up in the training set and 13 cases in the validation set. Among various cardiac adverse events, angina pectoris recurrence ranked top with the highest frequency.

In this study, the results of univariate and multivariate analyses indicated that combined diabetes was a risk factor. The results of multivariate Cox regression analysis showed that patients with combined diabetes had a 4.269-fold (95% CI: 1.836–9.927) increased risk of disease progression after PCI. Relevant literature has also shown that the absolute risk of death is three times higher in diabetic patients than in nondiabetic patients [13]. Therefore, much attention should be paid to the continuous detection and control of blood glucose in patients with diabetes after PCI to control blood glucose within a reasonable range and reduce its damage to target organs, which in turn reduces the occurrence of cardiac adverse events and improves the quality of life of patients after surgery [14].

The results of this study showed that age was also an independent risk factor for cardio genesis 2 years after PCI, suggesting an increasing trend of incidence of cardiac adverse events with increasing age [15]. BMI also played a part in the occurrence of cardiac adverse events, and patients should be informed to pay attention to dietary habits and maintain healthy lifestyle. Moreover, attention should equally be paid to creatinine clearance rate and left ventricular ejection fraction at any time [16], and preventive measures should be taken as early as possible to forestall the deteriorating prognosis of patients.

In summary, this study constructed a risk model based on the clinical features of the CTO patients, which has a good performance for predicting the risk of disease progression after PCI, thus enriching the predictive means for the prognosis of patients in clinical practice. However, there are limitations in this study. For one thing, the sample size is small. Hence, more sample information needs to be included. For another, there is still room for the optimizing of this predictive model by considering the effect of other complications on disease progression, which may help to develop a more accurate prognostic prediction model, thereby reducing the incidence of short-term and long-term postoperative cardiovascular events.

## Figures and Tables

**Figure 1:** Nomogram of independent risk factors predicting progression-free survival in patients with CTO. Notes: each patient's age, BMI, diabetes, and other 5 indicators in this nomogram have a corresponding score, and the sum of these scores corresponds to the total points. The total points correspond to 1-year disease progression rate and 2-year disease progression rate, respectively.

**Figure 2:** Internal and external validation.

**Figure 3:** Internal and external validation.

**Table 1:** Comparison of baseline information of patients.

Baseline information	Training set (*n* = 54)	Validation set (*n* = 28)	*p* value
Age			0.941
≤57	27	15	
>57	27	13	
Sex			0.796
Male	22	13	
Female	32	15	
BMI	24.74 ± 3.40	24.68 ± 2.77	0.351
Smoking history			0.572
No smoking history	16	11	
Smoked but quitted	20	8	
Still smoking	18	9	
Creatinine clearance rate	67.69 ± 10.29	67.89 ± 8.99	0.303
Left ventricular ejection fraction < 40%	44.65 ± 5.96	43.04 ± 5.43	0.359
Peripheral vascular disease	15	8	1.000
COPD	3	4	0.355
Hypertension	20	8	0.602
High cholesterol	5	4	0.750
Diabetes	12	5	0.861
Familial genetic history	8	4	1.000

**Table 2:** Univariate Cox regression analysis.

Factors	Hazard ratio	95% CI	*p* value
Age	1.086	1.035-1.139	<0.001
BMI	1.102	0.999-1.215	0.052
Sex	1.544	0.679-3.511	0.300
Smoking history	0.977	0.589-1.618	0.927
Creatinine clearance rate	0.954	0.916-0.993	0.022
Left ventricular ejection fraction	0.860	0.793-0.931	<0.001
Peripheral vascular disease	1.420	0.610-3.306	0.416
Hypertension	0.707	0.303-1.648	0.422
High cholesterol	0.799	0.188-3.395	0.761
Diabetes	4.269	1.836-9.927	<0.001
Familial genetic history	0.178	0.024-1.324	0.092

**Table 3:** Multivariate Cox regression.

Factor	Hazard ratio	95% CI	*p* value
Age	1.113	1.023-1.092	0.006
BMI	1.290	1.081-1.440	<0.001
Diabetes	2.873	0.916-9.685	0.047
Creatinine clearance rate	0.935	0.899-0.987	0.008
Left ventricular ejection fraction	0.857	0.781-0.924	<0.001

## Data Availability

The data used to support the findings of this study are available from the corresponding author upon request.
